RETRACTED

# Path of Regional Economic Transformation and Upgrading Based on Recurrent Neural Network

**DOI:** 10.1155/2022/1547837

**Published:** 2022-05-31

**Authors:** GuoJun Liang, Aiping Zhao, Xueshuang Xin

**Affiliations:** ^1^School of Economics and Management, Shijiazhuang University, Zhufeng Street, Yuhua District, Shijiazhuang 050035, Hebei, China; ^2^School of Literature and Media, Shijiazhuang University, Zhufeng Street, Yuhua District, Shijiazhuang 050035, Hebei, China

## Abstract

At present, the development of the regional economy is very rapid and widespread. However, due to increasingly prominent problems such as the low level of technological innovation and the unreasonable industrial structure, the economic growth rate has declined. Therefore, it is particularly important to use the circular economy network to study the transformation and upgrading of the regional economy. It clarifies the stakeholders in the process of transformation and upgrading of manufacturing enterprises. Its benefits in the network are given, and symptoms and mobilization methods and the obstacles and solutions to the development of mobilization among various subjects are drawn. In addition, it also emphasizes the equivalence between intelligent products and human subjects in this network. Because of the intelligence carried by products under the current background, diversified connotations and functions are becoming more and more abundant. The empirical results show that the pulling coefficients of residents' consumption level, the development of modern service industry, and urbanization rate to economic growth are 0.1812, 0.7165, and 0.1635, respectively, while the pulling coefficient of Gini coefficient to economic growth is −0.1785.

## 1. Introduction

Under the new normal, the high consumption, high investment, and low-efficiency economic growth model in the past can no longer meet the requirements of today's social development. How to maintain healthy and sustainable economic development is the main issue facing China's economy. At the same time, due to the different economic bases among different regions in China, the level of technological innovation and the development of industrial structure are unbalanced. Therefore, the level of economic development between regions has gradually increased. It enhances the level of technological innovation and promotes the transformation and upgrading of the industrial structure, so as to achieve coordinated development between regions in China. This is of great strategic significance to the transformation of China's economic structure and the realization of a moderately prosperous society in an all-around way.

Regional economics, as a discipline that studies the development law of “economic regions” and the occurrence and development of spatial differences, is different from microeconomics, which studies elements. It is also different from macroeconomics, which studies the national economy. Instead, it targets administrative regions of a specific scale and applies the viewpoints of various disciplines such as economics and geography. It studies the development and changes in the regional economy and promotes regional economic development. Facing the research on the laws of regional transformation and related issues that are taking place under the impetus of economic globalization, this paper starts from the perspective of regional economics, seeking theoretical support and exploring the path of transformation to enrich the subject content. It is of great significance to the research on the new problems of spatial pattern and the development of disciplines brought about by the promotion of regional development. This paper analyzes and judges the path of regional transformation and predicts the situation and direction of future development.

RETRACTED

The innovations of this paper are as follows. (1) In the process of researching enterprise transformation, it is based on the internal transformation of the enterprise, and this thesis focuses on the current comprehensive competitive advantage of the enterprise. (2) This paper is based on the macro perspective of internal and external relations of enterprises, using value chain theory and actor-network theory. It places manufacturing enterprises in a complete ecological network to study their transformation and upgrading mechanisms, and it analyzes their transformation and upgrading paths. (3) It raises the logic of “Internet + manufacturing” to the level of the whole value chain of enterprises, and it studies the path of Internet thinking to promote the transformation and upgrading of manufacturing enterprises.

## 2. Related Work

The development trend of regional economic transformation is becoming more and more intense, so many researchers have carried out research on it. Among them, Tachia and Ren-Huai illustrated some key management issues and challenges in specific contexts faced by countries and enterprises in terms of strategy and innovation during China's socioeconomic transition from various perspectives. The results demonstrate a broad range of aspects and diverse perspectives, demonstrating some key management issues and context-specific phenomena relevant to contemporary Chinese strategy and innovation development [1]. Islam and Ghosh showed that the economic transformation of the Indian state of West Bengal is reflected in an increase in occupational diversification. Per capita income increased, poverty levels decreased, and savings and loans decreased due to flooding [2]. To contribute to the key ontology of socioeconomic transformation processes, Bonifati discussed the possible development of the ontology of socioeconomic transformation processes. He came to the following conclusions. His contribution to this ontology was to show that the emergence of a new division of labor as a qualitative change requires a change in the relationship between the entities of the existing division of labor, giving it new functions and new directions [3]. In the context of transformational changes in the economic environment, the specific characteristics of informal employment have been identified and current trends are analyzed. The Bondarevska had confirmed the priority orientation of national policies aimed at eliminating threats from the informal labor market. The study highlights current trends in informal employment in the Ukrainian labor market [4]. Dalakian was devoted to the forming history of the Armenian diaspora in the Republic of Uzbekistan and its contribution to the socioeconomic transformation of the country. He cited the Armenian diaspora as an example, paying particular attention to the establishment and development of national cultural centers that promote indigenous cultures and traditions, as well as their historical home ties [5]. Prihatiningtyastuti argued that the participation of regional women in the structural transformation of Indonesia's economy has been challenged by cultural and structural factors. He analyzed reports, statistics, and previous work on women's participation and transition to formal employment. He found that Indonesian women's participation in the labor force and labor market is still lower than that of men [6]. Although there are many monetary and economic policies in the literature that were formulated before and after the new era in Zimbabwe, the country is still facing a downward trend in terms of economic recovery. Mazhazhate et al. reviewed the various policies implemented by the government and their impact on the socioeconomic development of Zimbabwe. The country has fallen from one of the best economies in sub-Saharan Africa to now struggling. It is characterized by hyperinflation, agricultural challenges, corruption, high taxation system, huge debt, consumers increasing prices, and becoming a major net importer of most goods or services [7]. While the research was supported by a case study survey of Singapore's renaissance, qualitative and quantitative tools were not used.

RETRACTED

## 3. Regional Economic Transformation Method of Recurrent Neural Network

### 3.1. Mechanism of Industrial Structure Transformation and Upgrading and Economic Growth

The rationalization of industrial structure refers to the adjustment of industrial structure in a certain stage of economic development, according to the level of science and technology, the structure of consumer demand, the basic quality of the population, and resource conditions, so that it can reach a reasonable state. That is, the various production factors can be reasonably allocated, and coordinated development between industries can be achieved [8, 9]. That is to say, the rationalization of industrial structure can strengthen the cohesion among various industries. This cohesion is not simply summing up various industries but will form a spillover effect [10, 11]. The level of this cohesion also determines how much the rationalization of the industrial structure can promote economic growth. The higher the cohesion force and the lower the cohesion force means that the factors of production cannot flow reasonably between industries. It shows that the higher the efficiency of the allocation of various production factors, the stronger the linkage between various industries, and the production efficiency of various industries is greatly improved, thereby promoting the improvement of total social output. It may have problems such as overcapacity in some industries, and the production efficiency will be greatly reduced, thus hindering economic growth [12, 13]. The shape of the three industrial economies is shown in Figure 1.

As shown in Figure 1, the advanced industrial structure refers to the dynamic process of the industrial structure changing from a low-level form to a high-level form, that is, from the primary industry to the secondary and tertiary industries [14, 15]. When the industrial structure is relatively low level, the output is mainly labor-intensive products. With low added value and low production efficiency, when the industrial structure gradually turns to an advanced form, labor-intensive industries are gradually replaced by technology-intensive industries. This product is characterized by a low level of technology, and some high value-added, high-tech products are produced. It has greatly improved social production efficiency, and these technology-intensive industries have also begun to become new engines of economic growth [16].

### 3.2. Recurrent Neural Network Algorithm

The relationship between input and output in the investment problem is nonlinear. Artificial neural networks utilize a combination of linear relationships in multiple layers of internal neurons, which can well approximate nonlinear relationships [17–20]. This section proposes an improved BPANN method, which attempts to use nonlinear mapping inside the artificial neural network to simulate the relationship between input and output.

RETRACTED

#### 3.2.1. BP Algorithm

The BP algorithm is a supervised learning artificial neural network [21, 22]. Its structure uses the steepest descent method or its improved algorithm to continuously update the network weights, so as to achieve a higher-precision approximation [23]. The usual structure of the BP algorithm is shown in Figure 2.

As shown in Figure 2, on this basis, the backpropagation algorithm of the multilayer neural network is improved, that is, the BP neural network model [24, 25]; let

(1) $$\begin{array}{c} \text{net}=\sum_{i=1}^{n}w_{i}x_{i}+b. \end{array}$$

Let *y* be the output of the network and let *f*_*h*_ be the system excitation function, i.e.,

(2) $$\begin{array}{c} y=f_{H}\left(\text{net}\right). \end{array}$$

Generally, the excitation function is taken as the sigmoid function:

(3) $$\begin{array}{c} f_{H}\left(\text{net}\right)=\log\text{sig}\left(\text{net}\right)=\frac{1}{1+\exp\left(-\text{net}\right)},\\ \text{or }f_{H}\left(\text{net}\right)=\tan\text{sig}\left(\text{net}\right)=\frac{1-\exp\left(-\text{net}\right)}{1+\exp\left(-\text{net}\right)}. \end{array}$$

Let

(4) $$\begin{array}{c} O=f_{o}\left(y\right). \end{array}$$

It is the excitation function of the output unit, usually selected as a linear function; this paper selects

(5) $$\begin{array}{c} O=f_{o}\left(y\right)=y=f_{H}\left(\text{net}\right). \end{array}$$

The mean square error (MSE) is the sum of the squares of the true value and the network output value:

(6) $$\begin{array}{c} \text{MSE}=\frac{1}{N}\sum_{i=1}^{N}{\left(\text{true}-\text{output}\right)}^{2}. \end{array}$$

In investment decision-making, true represents the output value obtained through investment, and output represents the continuous training of the BP network.

The final output value obtained by training, *N* represents the capacity of training samples [26]. The designed BP algorithm is to minimize MSE through continuous training of samples, that is, to form the following optimization problem:

(7) $$\begin{array}{c} \min\frac{1}{N}{\sum_{j=1}^{N}\left(g_{j}-f_{j}\left(\sum_{i=1}^{n}w_{i}x_{i}+b\right)\right)}^{2}\\ \text{s.t}w_{i}\in \left[0,1\right]\left(i=1,i=2,\ldots ,n\right),\;b\in R. \end{array}$$

#### 3.2.2. Improved BP Model

Consider the following questions, and the investment and output table is shown in Table 1.

As shown in Table 1, *Y*(*i* = 1,2,…, *s*) represents the year, and A_nn_ represents the investment of the jth industry in the ith year. *g* (*i* = 1,2,…, *s*) represents the output in year *i*. It writes the structure of the network as a map:

(8) $$\begin{array}{c} f\left(w_{1}{\vec{a}}_{1}+w_{2}{\vec{a}}_{2}+w_{3}{\vec{a}}_{3}+b\right)=\vec{g}. \end{array}$$

Among them,

(9) $$\begin{array}{c} f\left(t\right)=\log\;sig\left(t\right),\\ \text{or }f\left(t\right)=\tan\;sig\left(t\right), \end{array}$$

*w*_*i*_ ∈ [0,1](*i*=1, *i*=2,…, *n*) is the weight.

(10) $$\begin{array}{c} {\vec{a}}_{1}=a_{ji}\left(i=1,2,\ldots ,s\right). \end{array}$$

It is an investment vector:

(11) $$\begin{array}{c} \vec{g}=g_{j}\left(j=1,2,\ldots ,s\right). \end{array}$$

It is the total output value vector. In this way, the investment decision problem can be written as an optimization problem as follows:

(12) $$\begin{array}{c} \min\frac{1}{N}\sum_{j=1}^{N}\left(\left(g_{j}-f_{j}w_{1}{\vec{a}}_{1}+w_{2}{\vec{a}}_{2}+w_{3}{\vec{a}}_{3}+b\right)\right)\\ \text{s.t}w_{i}\in \left[0,1\right]\left(i=1,i=2,\ldots ,n\right),\;b\in R. \end{array}$$

The optimization problem in the above artificial neural network is to perform nonlinear mapping on the linear superposition of the three industrial investments to realize the nonlinear functional relationship between the overall gross output value and each industry. This nonlinear mapping can be improved by noting the nonlinear relationship between gross output value and each industry, supposing

(13) $$\begin{array}{c} b=b_{1}+b_{2}+b_{3}. \end{array}$$

Converting the ternary linear form of the function arguments in formula (13),

(14) $$\begin{array}{c} w_{1}a_{j1}+w_{2}a_{j2}+w_{3}a_{j3}+b. \end{array}$$

Rewrite it as

(15) $$\begin{array}{c} \left(w_{1}a_{j1}+b_{1}\right)+\left(w_{2}a_{j2}+b_{2}\right)+\left(w_{3}a_{j3}+b_{3}\right). \end{array}$$

Thus, the above optimization problems (14) and (15) are transformed into the following form:

(16) $$\begin{array}{c} \min\frac{1}{s}{\overset{N}{\underset{j=1}{\sum }}\left(g_{j}-f\left(w_{1}a_{j1}+b_{1}\right)+\left(w_{2}a_{j2}+b_{2}\right)+\left(w_{3}a_{j3}+b_{3}\right)\right)}^{2}\\ \text{s.t}w_{i}\in \left[0,1\right]\left(i=1,i=2,\ldots ,n\right),\;b\in R. \end{array}$$

In order to more clearly reflect the nonlinear relationship between the total output value and the investment of various industries in the artificial neural network, it changes the original linear relationship between the neurons in the artificial neural network. It seeks to replace the linear form of the above optimization problem with a nonlinear function *u*(*a*):

(17) $$\begin{array}{c} w_{1}{\vec{a}}_{1}+w_{2}{\vec{a}}_{2}+w_{3}{\vec{a}}_{3}+b. \end{array}$$

The setting of the nonlinear function should conform to the nonlinear relationship between the total output value and the investment of various industries.

RETRACTED

## 4. Experiments and Path of Regional Economic Transformation and Upgrading

Among the many literature studies on the measurement of economic transformation, the regional economic transformation index system has not been unified, and the measurement methods are mostly judged by one or two. On the basis of fully absorbing the literature results, this paper constructs an evaluation system for regional economic transformation and uses a combination of methods such as principal component analysis, cluster analysis, and spatial differentiation. The regional economic transformation is measured and evaluated from multiple levels and multiple scales. The specific measurement ideas are shown in Figure 3.

As shown in Figure 3, the evaluation scale includes regional scale and city scale, and the analysis level includes comprehensive score evaluation and spatial differentiation evaluation. The evaluation scale includes regional scale and city scale, and the analysis level includes comprehensive score evaluation and spatial differentiation evaluation. The comprehensive evaluation is obtained by the principal component analysis method. It examines the development index and the adjustment index, respectively, according to the correlation between the original data, and it finally forms the evaluation of the comprehensive score of the transformation; the differential evaluation is based on the index system and the comprehensive evaluation. It adopts the spatial differentiation method to analyze the global spatial pattern and local spatial pattern of economic transformation.

### 4.1. Setting of Transformation and Upgrading Indicators

The demand structure includes domestic demand and external demand. Domestic demand includes consumption and investment. External demand is export. Economic growth is mainly driven by investment, consumption, and export. People call it the “troika.” The traditional development model has caused an imbalance in China's demand structure with overinvestment and underconsumption. The coordinated growth of consumption and investment is conducive to the healthy and sustainable development of the economy. However, China's current demand structure is long-term incoordination between the two. The low consumption rate of residents has led to the overall consumption rate being lower than the investment rate. This has resulted in excess production capacity in China and an imbalance in the structure of commodity supply and demand. The main reason for the imbalance of China's national economic system is that the consumption rate has been seriously lower than the consumption rate required for endogenous economic growth; that is, the contribution rate of domestic demand to the economic growth rate is too low. Combining the above viewpoints, it can be concluded that the traditional economic development method focuses on investment and export, while consumption is in a downturn. According to the National Bureau of Statistics, in 2013, the contribution rate of Chinese residents' consumption expenditure to GDP was 36.17%, which was far lower than the world average of 70%–80%. Therefore, this paper uses the household consumption rate to quantify the demand structure and analyze its relationship with economic growth. It applies the causal relationship test between InIGDPr, InCon, lnMsr, InUr, and InGcr. When the lag period is 2, the final test results are shown in Table 2.

RETRACTED

It can be seen from the test results in Table 2 that InCont and InGct are the reasons for the Granger causality of lnIGDPr at the 5% significant level. At the 10% significance level, InMsr and lnUr are responsible for the Granger causality of lnIGDPt.

### 4.2. Multiple Regression

In this paper, multiple linear regressions were performed on lnIGDP, InCon, InMsr, lnUr, and lnGc. InCon, InMsr, lnUr, and lnIGDP were positively correlated, and InGc was negatively correlated with InIGDP. Specifically, for every 1 percentage point increase in the household consumption rate, the economic growth index will increase by 0.1812 percentage points. For every 1 percentage point increase in the urbanization rate, the economic growth index will increase by 0.1635 percentage points; for every 1 percentage point increase in the proportion of modern service industry in GDP, the economic growth index will increase by 0.7165 percentage points. For every 1 percentage point increase in the Gini coefficient, the economic growth index decreases by 0.1785 percentage points.

Through empirical research on the relationship between economic growth and economic transformation and upgrading, the following important conclusions are drawn. First, the consumption level of Chinese residents, the development of the modern service industry, the development of cities and towns, and the size of the Gini coefficient are all reasons for driving economic growth. In order to overcome the “middle-income trap,” economic transformation and upgrading must balance the imbalances in demand structure, industrial structure, urban-rural structure, and income distribution structure from the level of residents' consumption, the development of modern service industry, urban development, and income distribution. Second, the consumption level of Chinese residents, the development of urban areas, and the level of service industry development can all drive economic growth. The higher the Gini coefficient, the more inhibiting the economic growth. The empirical results show that the pulling coefficients of residents' consumption level, the development of modern service industry, and urbanization rate to economic growth are 0.1812, 0.7165, and 0.1635, respectively. The pull coefficient of the Gini coefficient to economic growth is −0.1785. Therefore, China must improve the consumption level of residents and the development level of the service industry. It vigorously promotes urbanization. It also reduces the Gini coefficient by adjusting the income distribution structure. It is expected to further promote economic transformation and upgrading and overcome the “middle-income trap.”

RETRACTED

## 5. Path of Regional Economic Transformation and Upgrading

Under the background of “Internet +,” manufacturing enterprises need to build a holistic and global value chain. In this value chain, there are consumers, partners, and suppliers through collaborative efforts, so that each subject can obtain corresponding benefits from it. Then, the construction of the value chain can be reconstructed from an overall perspective, which is the purpose of maximizing benefits through resource integration on the basis of the original value chain. Therefore, relying on the “Internet +,” manufacturing enterprises can rely on their own advantages to obtain higher-income parts of the value chain. Once it chooses a path that is in line with itself for transformation, it can go beyond the development of the conventional model and obtain the greatest benefits. Under the new normal, manufacturing enterprises must learn to use the thinking of “Internet + manufacturing” to rationally optimize resources. It uses “Internet +” to improve the level of informatization, develop intelligent manufacturing, and integrate value chain functions. It realizes strategy and management innovation and promotes the transformation and upgrading of manufacturing enterprises.

### 5.1. Manufacturing-Intelligent Manufacturing Based on Internet and Big Data

Intelligent manufacturing is an integration of human and machine resources, and the fusion of information and manufacturing technology, which facilitates automated production. It is an efficient production method from self-diagnosis to self-execution. Effectively different from the rigid mode of traditional production, the production of intelligent manufacturing has the characteristics of flexibility. In the industrial Internet, products with sensors and other properties are effectively connected to machines and equipment. It is continuously optimizing the performance of various indicators of the machine with the help of software analysis. In a smart workshop, different machines and different equipment can cooperate efficiently. In this way, the entire intelligent workshop can operate dynamically and finally achieve an efficient production operation mode in order to reduce consumption. At the factory level, relevant personnel will optimize and adjust between various production lines and different workshops when fully combining production tasks according to the actual situation of the current market and supply chain. In order to optimize the cooperation between humans and machines, it achieves this goal by changing the performance of machines and equipment based on improving the efficiency of people through various types of equipment and connection methods. It can be said that this is a systematic project. Through the transformation of the original low-end value chain to the high-end value chain, it will finally achieve a successful upgrade of the enterprise.

RETRACTED

Through the combination of the Internet, computers, and open hardware platforms, users' design thinking and process concepts for smart products can be transmitted to enterprises in a timely manner. It will become possible to gather the wisdom of all people, meet the needs of users, and make it by itself. The production chain of individual production appears in front of people. It leads the manufacturing industry toward decentralization and flat development. Facts have proved that many manufacturing enterprises have gained development advantages from it. It carries out private customization activities guided by consumer demand and achieves the purpose of small-scale batch production. Among them, Haier and Xiaomi have successful experience in this regard. So, in the near future, everyone will have their own personalized customized products, which will no longer be a distant dream. The R&D model of manufacturing enterprises driven by “Internet +” is shown in Figure 4.

As shown in Figure 4, if manufacturing companies want to break through technical barriers and quickly realize technological leaps and upgrades, they must pay attention to the power of the maker movement and consumers. This paper believes that the R&D model of manufacturing enterprises should be transformed from a single enterprise internal R&D or directional cooperative R&D to a micro-R&D system of makers + consumers. It cooperates with the innovative research and development of the scientific research alliance. Only in this way can it break the vicious circle that was originally dominated by large enterprises in the industry to achieve new technology breakthroughs.

### 5.2. Organizational Structure to Meet Organizational System Reform of Dual Management Capabilities

Driven by the “Internet +,” the organizational system of manufacturing enterprises has undergone profound changes. The traditional bureaucratic connection mode gradually decomposes, and the network-like connection cycle mode gradually emerges. In the future, the interior of manufacturing enterprises will be in the form of “networking, modularization, and informatization.” However, the network organization system is not disordered but differentiated and integrated according to functional modules to form a functional network structure. It includes a decision-making organization system, research and development organization system, production organization system, and market organization system. Among them, the decision-making organization system provides major decision-making functions for enterprise development, such as development goals, development plans, and development policies. The R&D organization system provides R&D support for technological upgradings, such as common technologies and key technological breakthroughs. The production organization system opens up the product, such as the product opening up the road of intelligent manufacturing and technology deconstruction and integration. The market organization system provides functions to solve the contradiction between supply and demand, such as the establishment of market platforms and the dredging of information channels. All organizational systems are interconnected, forming an open loop. The analysis of the organizational structure upgrade mode of manufacturing enterprises based on functional modules is shown in Figure 5.

RETRACTED

As shown in Figure 5, with the rapid development of the mobile Internet, e-commerce has accelerated the deep integration of local and international development, which means that consumers' needs will be more diversified. For manufacturing enterprises, the organic combination of high-standard products produced by consumer demand-oriented production and high-quality services can continuously expand their business scope. In this regard, the organizational structure of manufacturing enterprises will be transformed, and collaborative production will become its development trend. The decision-making organization system, R&D organization system, production organization system, and market organization system of each enterprise can also be connected with the corresponding organizational function systems of other enterprises. It uses the borderless characteristics of the Internet to achieve information exchange and resource sharing. This is consistent with the connotation of the concept of intelligent alliance mentioned earlier. Relying on the Internet, all links in the manufacturing industry and the people in each link have become communicators of information, which will greatly improve communication efficiency with the help of modern communication software. This lays the foundation for improved work efficiency. In essence, the formulation of strategies in the manufacturing industry is fundamental to enhancing comprehensive competitiveness. In order to expand its own competitiveness, it will adopt a variety of methods for collaborative production.

RETRACTED

### 5.3. Strategic Decision-Making Shift from Internal Division of Functions to Internal and External Collaboration

The purpose of efficient management is to ensure that the organization achieves the purpose of rapid operation through collaborative division of labor. When an enterprise's execution is stronger, it can show that the enterprise has the best collaborative division of labor. When this division of labor can effectively solve various problems in the organization, such management is more effective, so that a new realm of synergy can be achieved. Connection is one of the essences of “Internet +.” The connection here includes not only the connection between various functional departments and business processes within the enterprise but also the connection between the enterprise and the outside world. Internal and external collaborative manufacturing is extended from the inside out according to the depth of application of the enterprise. The first is the collaboration based on the internal workflow of the enterprise, which covers all employees based on forms, approvals, etc. It also extends to integration with business systems. It then integrates and collaborates based on unified platform architecture, breaking the boundaries of products in various fields. This ensures a high degree of collaboration between the various segments. This high degree of collaboration enables dynamic and intensive management between different organizational departments and different regions. At the same time, it uses the Internet as a medium to strengthen the exchange of information and form a complete set of knowledge system management. This lays the foundation for ensuring the smooth running of the organization. The static tests performed in this section take the form of unit root ADF tests and are performed using EViews 6 software. The test results of variable stationarity are shown in Table 3.

According to the test results in Table 3, it can be known that the selected three variables are stationary in the horizontal series. The ADF statistics are all below the 5% critical value, so the time series data of these three variables are stationary series. Such an organizational structure system can be properly controlled from vertical management to horizontal detailed control. In this way, the flexible management of the organization is more in place. On the basis of internal connectivity, manufacturing enterprises also need to gradually expand outward to form good interactions with various groups in the value chain. At the same time, it can form an integrated management purpose between virtual organization management and entity organization management. For social collaboration, corporate boundaries are becoming increasingly blurred. They need to integrate the upstream and downstream resources of the industrial chain and build a synergy based on the industrial chain. It connects the internal organization of the enterprise with the external organization. Ultimately, it is social collaboration, which integrates resources from all parties, so that enterprises can become more smooth in social collaboration and business flow. For example, the positions set up in some enterprises are similar to such “post mailboxes,” and these jobs will be handled by special personnel, and the information will be collected centrally. It also conducts a unified comparison and analysis based on the collected information and finally transmits this effective value information through various mobile platforms. In the end, someone will provide unified feedback on this kind of information. The purpose of this is to communicate all kinds of external information and then process them internally to strengthen the collaborative processing of information. The reduction is due to changes in results due to problems in the communication and processing of internal and external information. The scatter diagram of the relationship between regional cultural industry development and economic transformation and upgrading ability, technological innovation investment and economic transformation and upgrading ability, human capital and economic transformation and upgrading ability, foreign investment scale and economic transformation and upgrading ability, and professional market scale and economic transformation and upgrading ability are as shown in Figures 6 and 7.

RETRACTED

From the scatter plots in Figures 6 and 7, it can be seen that the development of the cultural industry and the ability of economic transformation and upgrading have obvious characteristics of codirectional changes. That is, the development of the cultural industry has a positive impact on the transformation and upgrading of the regional economy. The development of the cultural industry promotes the transformation and upgrading of the regional economy. Technological innovation investment, human capital, foreign investment and professional market scale, and economic transformation and upgrading capabilities also have obvious comovement characteristics. This shows that technological innovation ability, human capital, foreign investment scale, and market environment have a positive role in promoting regional economic transformation and upgrading. Next, this chapter examines and reveals the relationship between cultural industry development, technological innovation input, human capital, foreign investment, specialized market size, and economic transformation and upgrading capabilities from a regional level through quantitative analysis.

Enterprises with great development prospects are good at using the Internet platform, oriented by customer needs and incorporating the needs of suppliers into the value chain. It obtains greater profit value space through the rational allocation of resources. In the context of global integration, enterprises rely on technologies such as big data to maximize value. This means that companies need to coordinate resources in all aspects. The business model has certain market development prospects, the warehouse design is relatively complete, the distribution business is relatively reasonable, and the business system operates more efficiently. While the system integrator provides top-level rules, it must also accept the module supplier's reform of the rules. It thus forms product technology innovation. The modular value chain integration of manufacturing enterprises is shown in Figure 8.

As shown in Figure 8, when the current changes in consumer demand show irregular characteristics, manufacturing enterprises will face the changing needs of customers and rely on the Internet platform to achieve greater development. At the same time, manufacturing enterprises can create platforms and open them to various entities based on products. Each participant can combine their own capabilities to develop and produce products. It further shortens the life cycle of products and ultimately meets the needs of customers to generate revenue. The modular integration between manufacturing enterprises (industries) is shown in Figure 9.

As shown in Figure 9, on the basis of the modular integration of the value chain, manufacturing enterprises should fully consider and understand their main competitiveness. It then analyzes the product audience and subsequent research and development work. After understanding these links, it finally chooses Internet tools suitable for the development of the enterprise itself and reconstructs the business model.

## 6. Conclusion

China's industrial structure has long been overcapacity in some industries, and some industries cannot be effectively supported due to limited resources. There is a phenomenon of high-tech content and few high-value-added products in the manufacturing industry, so an effective elimination mechanism must be established. It will eliminate outdated production capacity and allocate resources to industries with low consumption, less input, and higher output efficiency. In addition, the optimization of industrial structure is inseparable from the support of high-quality talents. Therefore, China should improve the talent training mechanism and establish a training system for different types of talents to match the development needs of various industries. It promotes the rational flow of talents in various industries. It reduces the structural unemployment problem in the labor market so that human resources can be maximized. It promotes industrial development and economic growth. It adapts measures to local conditions and reasonably promotes the upgrading of the industrial structure. The essence of the advanced industrial structure is the service-oriented tendency of the economic structure; that is, the proportion of the tertiary industry in the economic structure occupies a major position. China is also facing the stage of transition from manufacturing to the service industry at this stage, so the advanced industrial structure is also the main problem facing China. However, the goal of the advanced industrial structure is not only to expand the output value of the tertiary industry but also to integrate and develop with other industries toward the service-oriented trend of the economic structure. This integration model not only improves the efficiency of industrial output but also can effectively improve the quality of economic development. The producer service industry is a link between the secondary industry and the tertiary industry. This paper vigorously enhances the support for producer services and, through this connection, deepens the division of labor in the industrial chain. It continuously promotes the interaction between industries and realizes the advanced development of the industry. In addition, in recent years, China has proposed vigorously developing emerging strategic industries and service industries. Various regions have actively responded to the national call and issued a series of policies and measures to promote the development of the service industry, but the economic development level gap between regions in China is relatively large. The level of economic development in some regions is still at a relatively low stage and blindly follows. Instead of adjusting the industry according to local conditions, it is not conducive to economic growth. There are still some areas that need to be improved in this paper; first of all, the selection of indicators needs to be improved. For the selection of technical innovation indicators, this paper selects indicators that can measure the level of technical innovation under the premise of data availability. However, because the content of technological innovation is too broad, the selected indicators cannot fully reflect the level of technological innovation, so the relevant empirical relationship needs to be further improved.

RETRACTED

## Figures and Tables

**Figure 1:** The form of the three industrial economies.

**Figure 2:** The structure of the artificial neural network.

**Figure 3:** The specific measurement ideas for the measurement and evaluation of regional economic transformation.

**Figure 4:** The R&D model of manufacturing enterprises driven by “Internet +.”

**Figure 5:** Analysis of the organizational structure upgrade mode of manufacturing enterprises based on functional modules.

**Figure 6:** Scatter diagram of cultural industry development, technological innovation, and economic transformation. (a) Scatter diagram of cultural industry development and economic transformation. (b) Scatter diagram of technological innovation and economic transformation.

**Figure 7:** Scatter plot of human capital, size of foreign capital and specialized markets, and economic transformation. (a) Human capital economic transformation. (b) The scale of foreign investment and economic transformation. (c) Scatter plot of specialized markets and economic transformation.

**Figure 8:** Modular value chain integration of manufacturing enterprises.

**Figure 9:** Modular integration between manufacturing enterprises (industries).

**Table 1:** Investment and output table.

year	Invest			Gross output value
	Primary industry	Secondary industry	Tertiary industry	
Y_1_	*A*_11_	*A*_12_	*A*_13_	*g*_1_
Y_2_	*A*_21_	*A*_22_	*A*_23_	*g*_2_
…	…	…	…	…
…	…	…	…	…
*Y*_s_	*A*_s1_	*A*_s2_	*A*_s3_	*g*_*s*_

**Table 2:** Granger causality test.

Null hypothesis	F Statistic	Accompanying probability value	In conclusion
Reason for InCon, not InIGDP	3.73104	0.0489^*∗∗*^	Reject
lnIGDP is not an InCon the reason	0.76429	0.5009	Accept
InMsr, not the cause of lnIGDP	0.18142	0.0837^*∗∗∗*^	Reject
Reason for InIGDP not InMsr	1.57299	0.2728	Accept
InUr, not the reason for InIGDP	3.65465	0.0819^*∗∗∗*^	Reject
Reason for InIGDP not InUr	0.89609	0.4503	Accept
InGc, not the cause of InIGDP	0.49783	0.0427^*∗∗*^	Reject
Reason why InIGDP is not InGc	2.11052	0.1917	Accept

*Note.* ^*∗*^ means significant at 1% level; ^*∗∗*^ means significant at 5% level, ^*∗∗∗*^ means significant at 10% level.

RETRACTED

**Table 3:** Stationarity test of variables.

Variable	lnY	InK	InL
ADF statistic	−3.384889	−5.072700	−3.790854
Threshold (1%)	−3.670170	−3.699871	−3.639407
Threshold (5%)	−2.963972	−2.976263	−2.951125
Threshold (10%)	−2.621007	−2.627420	−2.614300
Is it stable	Smooth	Smooth	Smooth

## Data Availability

The data that support the findings of this study are available from the corresponding author upon reasonable request.

## References

[1] Tachia C., Ren-Huai L. (2017). Critical management issues in China’s socio-economic transformation. *Chinese Management Studies*.

[2] Islam A., Ghosh S. (2021). Economic transformation in the wake of flood: a case of the lower stretch of the Mayurakshi River Basin, India. *Environment, Development and Sustainability*.

[3] Bonifati G. (2020). Towards a critical ontology of socio-economic transformation processes: marx’s contribution. *Cambridge Journal of Economics*.

[4] Bondarevska K. V. (2020). Informal employment as a threat to social security in the labor market in Ukraine within an economic transformation. *The Problems of Economy*.

[5] Dalakian J. (2020). History of formation of the Armenian diaspora in Uzbekistan and its contribution to the socio-economic transformation of the country. *Bulletin of Science and Practice*.

[6] Prihatiningtyastuti E. (2020). Regional women’s economic participation: a systematic-based review of structural economic transformation in Indonesia. *Wawasan Jurnal Ilmiah Agama dan Sosial Budaya*.

[7] Mazhazhate C., Mujakachi T. C., Munuhwa S. (2020). Towards pragmatic economic policies: economic transformation and industrialization for revival of Zimbabwe in the new dispensation era. *International Journal of Engineering and Management Research*.

[8] Ma G. (2019). Analysis of economic transformation capacity and convergence of resource-regenerative cities—based on entropy weight TOPSIS method. *American Journal of Industrial and Business Management*.

[9] Wisesa O., Andriansyah A., Ibrahim Khalaf O. (2020). Prediction analysis for business to business (B2B) sales of telecommunication services using machine learning techniques. *Majlesi Journal of Electrical Engineering*.

[10] Tavera Romero C. A., Castro D. F., Ortiz J. H., Khalaf O. I., Vargas M. A. (2021). Synergy between circular economy and industry 4.0: a literature review. *Sustainability*.

[11] Habarta A. (2019). Double anniversary in Poland: 30 years of socio-economic transformation and 15 years of membership in the EU. *Contemporary Europe*.

[12] Atkinson R. D., Andes S. M. (2017). The 2010 state new economy index: benchmarking economic transformation in the states. *Social Science Electronic Publishing*.

[13] Strohmaier R., Schuetz M., Vannuccini S. (2019). A systemic perspective on socioeconomic transformation in the digital age. *Journal of Industrial and Business Economics*.

RETRACTED

[14] Mavesera M., Magege D. (2020). Fostering posterity and socio-economic transformation through the prism of indigenous languages in youth training: a participatory approach. *Southern Africa Journal of Education Science and Technology*.

[15] Dobrzyńska M. (2019). From technological revolution towards socioeconomic transformation – non-standard forms of job execution in the digital age. *Occupational Safety – Science and Practice*.

[16] Yin H. (2019). The development of the socialist market economy: practice of Chinese market economic transformation. *Humanities and Social Sciences Bulletin of the Financial University*.

[17] Pachkalov A. V. (2019). The development of the socialist market economy: practice of Chinese market economic transformation. *Humanities and Social Sciences Bulletin of the Financial University*.

[18] Alabbasi Y., Sandhu K. (2019). The framework for blockchain innovation and the impact on digital economic transformation. *International Journal of Innovation in the Digital Economy*.

[19] Khan A. N., Cao X., Pitafi A. H. (2019). Personality traits as predictor of M-payment systems: a SEM-neural networks approach. *Journal of Organizational and End User Computing*.

[20] Khalaf O. I., Romero C. A. T., Azhagu Jaisudhan Pazhani A., Vinuja G. (2021). VLSI implementation of a high-performance nonlinear image scaling algorithm. *Journal of Healthcare Engineering*.

[21] Nagi Alsubari S., Deshmukh S. N., Alqarni A. A. (2022). Data analytics for the identification of fake reviews using supervised learning. *Computers, Materials & Continua*.

[22] Meng F., Cheng W., Wang J. (2021). Semi-supervised software defect prediction model based on tri-training. *Ksii Transactions On Internet And Information Systems*.

[23] Tuano P. A., Cruz J. (2020). Structural inequality in the Philippines oligarchy, (Im)mobility and economic transformation. *Southeast Asian Economies*.

[24] Alekseev A. V., Kuznetsova N. N. (2019). Russian capital investment dynamics as an economic transformation factor. *Вестник Российской академии наук*.

[25] Gorman E. (2019). High tech and high touch: headhunting, technology, and economic transformation. *Contemporary Sociology: Journalism Review*.

[26] Siddiqui K. (2019). Economic transformation of China and India: a comparative political economy perspective. *Asian Profile*.

